The article "Vibration Control of a Helicopter Rescue Simulator on a Flexible Base" was retracted in 2023. Reasons: signs of a paper mill; compromised peer review; unreliable results or conclusions.

# Vibration Control of a Helicopter Rescue Simulator on a Flexible Base

**DOI:** 10.1155/2022/7173421

**Published:** 2022-04-25

**Authors:** Shengye Wang, Haitao Wang, Wei Xiong, Guangfeng Guan

**Affiliations:** Naval Architecture and Ocean Engineering College, Dalian Maritime University, DaLian 116026, Liaoning, China

## Abstract

The vibration compensation control of a hovering helicopter rescue simulator mounted on a crane beam is studied in this research. A Stewart platform is used as the motion generator of the helicopter simulation cabin and the vibration compensation device of the beam, simultaneously. This study describes how the dynamic model of the Stewart platform with consideration of the beam vibration is established. To determine the interference of the Stewart platform motion control in the special application of a large component flexible base requiring large-scale movement, a hybrid vibration controller composed of a feed-forward compensation module and a PD (proportional-derivative) feedback control module is designed. The experimental results show that this method can effectively compensate for the beam vibration and improve the accuracy of the motion reproduction of a helicopter simulation cabin.

## 1. Introduction

A helicopter hovering rescue simulator is used for the training of lifeguards when implementing tasks under harsh sea conditions in a laboratory environment. The helicopter hovering rescue simulator is installed on a bridge crane and can move with the crane around the rescue pool. The rescue pool, also called the wave pool, is equipped with two wave balls on both sides to simulate the wave shapes of severe sea conditions, as shown in Figure 1. During a rescue task training process, the simulator simulates the hovering flight state of a helicopter under bad sea conditions, and the rescue crew on the simulator rescues the victims in the violent waves. The Stewart platform, as a motion-generating device simulating the hovering motion state of a helicopter, connects the bridge crane and the simulated cabin. Its motion accuracy determines the authenticity of the simulation effect. When the Stewart platform drives the simulated cabin to move, the bridge beam supporting the quality of the whole system produces strong vibrations, which significantly affects the accuracy of the end effector (cabin) of the Stewart platform and the proprioception of the crew during training. The problem described above is that a parallel robot with a flexible base can be classified as the vibration isolation field of the Stewart platform [1]. In this study, the Stewart platform not only acts as an isolator but also as a vibration source for the flexible base (bridge beam), simulating the hovering motion state of the helicopter, which is different from other applications of Stewart isolation [2, 3].

In the control strategy of the Stewart platform, in addition to the commonly used PID (proportional-derivative-integral) control [4, 5], adaptive control [6] and robust control [7] are also employed. After the desired trajectory of the platform is provided, these control strategies achieve the purpose of controlling the platform by controlling the expansion or output force of the driving device. However, the dynamics of each leg of the Stewart platform are affected by nonlinear forces, and the dynamic coupling of each leg makes it very difficult for the controller to tune the parameters of the task space. A decoupling control strategy can be used to overcome this problem and obtain better performance [8–11]. However, the existing decoupling strategy is only suitable for a proportional damping matrix vibration system, and it is not suitable for a Stewart platform, considering the dynamics of the flexible support base.

There are three main active vibration control technologies: variable structure control technology, pulse active damping technology, and supervisory control technology. Variable structure control technology [12–14] can effectively suppress the vibration of flexible parts by actively adjusting the damping and stiffness of the original structure by placing elements or materials with sensing and actuation functions inside the structure. However, this distributed layout not only reduces the reliability of the system but also has a poor control effect on large flexible parts. According to the vibration feedback information of the flexible base sensor, by adding an external excitation robot, pulse active damping technology [15–17] excites the robot to produce a vibration exactly opposite to that of the base and eliminate the original base vibration. This technology only needs to be applied to the system after the vibration is started and measured. Then, real-time system identification is carried out, and the natural frequency and damping ratio of the system are obtained. Supervisory control technology [18–20] collects the motion information of the end effector of the Stewart platform, feeds back the motion state of the end effector to the controller, and achieves the full closed-loop control of the actuator with a high-precision two-level fine-tuning system. This method requires an additional motion acquisition system, and the control accuracy is affected by the accuracy, response speed, and filtering algorithm of the motion acquisition system. When a flexible base like the helicopter hovering rescue simulator needs to move over a large range, it will also cause problems such as installation difficulty, decreased system reliability, and high measurement cost [21, 22].

The feedforward technology of vibration control [23] is widely used because it does not require any additional sensors or actuators and has strong adaptability to system changes. Input shaping technology [24, 25] produces a better performance than other feedforward technologies (Butterworth, notch), and it is the most representative. Input shaping avoids inducing vibration during command movement by convoluting the pulse sequence with the desired command. When the pulse sequence is selected properly, even in the case of modeling uncertainty, it is only necessary to obtain the basic characteristics of the natural frequency and the damping ratio of the relevant modes to effectively eliminate the residual vibration. This feedforward technology has a good effect on eliminating the residual vibration of the robot [26, 27], but it is difficult to deal with the vibration elimination in the process of continuous motion, except for the start and stop stages of the robot. In this study, based on the dynamics of the Stewart platform and a flexible beam, a new feedforward control method is designed. For a flexible base parallel robot, feedforward control and feedback control technologies are used for vibration control and end position control, respectively. By developing a hybrid controller composed of two control technologies, the decoupling strategy of vibration control is achieved, and the complexity of the required feedback controller can be reduced.

To determine the special application of the crane beam of a helicopter rescue simulator, which has large flexible parts, violent vibration, and a large range of motion, the dynamic modeling method of a Stewart platform considering flexible support and the model-based compensation control method are proposed.

The main contributions of this study are as follows:

1. A dynamic model with consideration of the flexible support beam is established.
2. A hybrid controller including feedforward control and feedback control is designed, and a good vibration compensation effect is achieved.

The remainder of this study is organized as follows: the vibration interference problem of the Stewart flexible base is described in Section 2. In Section 3, the basic principle of the antivibration controller is introduced, and the dynamic model of the Stewart platform with consideration of the beam vibration is established. The experimental verification of the model is presented in Section 4. The conclusion is presented in Section 5.

## 2. Vibration Caused by the Stewart Platform

The helicopter hovering rescue simulator includes a trolley, a Stewart platform, an electric winch, a bridge crane beam, and a helicopter simulation cabin, as shown in Figure 2. The helicopter simulator cabin, which has a size similar to that of a Sikorsky S-76C, can accommodate at least six crew members for rescue training. The Stewart platform works to simulate the hovering motion of the helicopter. The platform hangs upside down on the trolley and is supported by the bridge crane beam.

The process of rescue training is as follows: The rescue target arrives within a specified range of the wave pool. At this time, the wave balls begin to create bad sea conditions. Then, the rescue crew that drives the simulator moves above the rescue target by controlling the bridge crane beam movement. The lifeguard hangs on the electric winch to complete the rescue of the target. In the whole rescue process, the Stewart platform continues to simulate the vibration of the helicopter cabin as a real flight to ensure the authenticity of proprioception in the rescue process.

When the Stewart platform is activated, the beam that supports the entire weight of the rescue system creates a forced vibration excited by the real-time changing movement of the simulator.  Figure 3 shows the vibration of the beam during a training process. It can be seen that the vertical vibration (curve *Z*) of the beam is similar to a harmonic motion with a 0.3 m/s^2^ amplitude and a 6 Hz frequency. A clear vibration can be felt when standing on the beam. When the horizontal vibration (curve *X* and curve *Y*) is one order of magnitude smaller than the vertical vibration, the influence on the somatosensory systems of the trainers can be neglected. For this reason, the actual motion trajectory does not fully match the input trajectory as well, which is mainly the result of the vertical vibration of the beam. Therefore, it is necessary to reduce the inaccuracy caused by the vibration of the flexible base.

## 3. Methods

### 3.1. Dynamics Model

The structure parameters of the inverted Stewart platform are shown in Figure 4. The parameters include the radius of the upper hinge *R*_*a*_, the radius of the lower hinge *R*_*b*_, the spacing of the upper hinge on the short side *L*_*s*_, the spacing of the lower hinge on the short side *L*_*x*_, the median length of cylinder *L*, and the stroke of the electric cylinder *S*. According to the characteristics of the Stewart platform mechanism, the basic structure of the platform can be determined by finding the above six parameters. The upper platform is connected with the beam through the crane trolley, and the vertical displacement of the beam *X*(*t*) is consistent with the vibration displacement of the upper platform. The center of the upper hinge circle is selected as the coordinate origin of the static coordinate system *OXYZ*, the center of the lower hinge circle is selected as the coordinate origin of the dynamic coordinate system *pxyz*, and the center position of the platform is defined as the initial pose of the platform.

The coordinates of the six lower hinge points in the *pxyz* coordinate system are represented by a matrix *A*′

(1) $$\begin{array}{c} A^{\prime }=\left[\begin{array}{cccccc} Ra\cdot c\alpha & -Ra\cdot s\left(\frac{\pi }{6}-\alpha \right) & -Ra\cdot c\left(\frac{\pi }{3}-\alpha \right) & -Ra\cdot c\left(\frac{\pi }{3}-\alpha \right) & -Ra\cdot s\left(\frac{\pi }{6}-\alpha \right) & Ra\cdot c\alpha \\ -Ra\cdot s\alpha & -Ra\cdot c\left(\frac{\pi }{6}-\alpha \right) & -Ra\cdot s\left(\frac{\pi }{3}-\alpha \right) & Ra\cdot s\left(\frac{\pi }{3}-\alpha \right) & Ra\cdot s\left(\frac{\pi }{3}-\alpha \right) & Ra\cdot s\alpha \\ -h & -h & -h & -h & -h & -h \end{array}\right], \end{array}$$

where *c* denotes the cosine, *s* denotes the sin, and *h* represents the height of the upper and lower platforms when the platform is in its initial position.

When the platform has an attitude *Q*=(*q*1,  *q*2,  *q*3,  *q*4,  *q*5,  *q*6), where *q*1 is the roll angle, *q*2 is the pitch angle, *q*3 is the yaw angle, *q*4 is the translation along the *px*, *q*5 is the translation along the *py*, and *q*6 is the translation along the *pz*, and the transformation matrix from coordinate *pxyz* to coordinate *OXYZ* is given by the following equation:

(2) $$\begin{array}{c} R_{P}=\left[\begin{array}{cccc} cq_{1}\cdot cq_{2} & cq_{1}\cdot sq_{2}\cdot sq_{3}-sq_{1}\cdot cq_{3} & sq_{1}\cdot sq_{3}+cq_{1}\cdot sq_{2}\cdot cq_{3} & q_{4}\\ sq_{1}\cdot cq_{2} & cq_{1}\cdot cq_{3}+sq_{1}\cdot sq_{2}\cdot sq_{3} & sq_{1}\cdot sq_{2}\cdot cq_{3}-cq_{1}\cdot sq_{3} & q_{5}\\ -sq_{2} & cq_{2}\cdot sq_{3} & cq_{2}\cdot cq_{3} & q_{6}\\ 0 & 0 & 0 & 1 \end{array}\right]. \end{array}$$

The matrix *A*′ can be written in the form of homogeneous coordinates as follows:

(3) $$\begin{array}{c} A=\left[\begin{array}{c} A^{\prime }\\ \left[\begin{array}{c} 1 \end{array}\right] \end{array}\right]. \end{array}$$

The coordinates of the six upper hinge points in the coordinate *pxyz* can be expressed in the static coordinate *OXYZ* with matrix **P** with the transformation matrix with *R*_*P*_, as follows:

(4) $$\begin{array}{c} P=R_{P}\cdot A. \end{array}$$

The coordinates of the six upper hinge points in the *OXYZ* coordinate system can be expressed as matrix B in the form of homogeneous coordinates, as follows:

(5) $$\begin{array}{c} B=\left[\begin{array}{cccccc} R_{b}\cdot c\left(\frac{\pi }{3}-\beta \right) & -R_{b}\cdot s\left(\frac{\pi }{6}-\beta \right) & -R_{b}\cdot c\beta & -R_{b}\cdot c\beta & R_{b}\cdot s\left(\frac{\pi }{6}-\beta \right) & R_{b}\cdot c\left(\frac{\pi }{3}-\beta \right)\\ -R_{b}\cdot s\left(\frac{\pi }{3}-\beta \right) & -R_{b}\cdot c\left(\frac{\pi }{6}-\beta \right) & -R_{b}\cdot s\beta & R_{b}\cdot s\beta & R_{b}\cdot c\left(\frac{\pi }{6}-\beta \right) & R_{b}\cdot s\left(\frac{\pi }{3}-\beta \right)\\ X\left(t\right) & X\left(t\right) & X\left(t\right) & X\left(t\right) & X\left(t\right) & X\left(t\right)\\ 1 & 1 & 1 & 1 & 1 & 1 \end{array}\right], \end{array}$$

where *X*(*t*) denotes the vertical displacement of the beam.

The length of the cylinder legs can be expressed as follows:

(6) $$\begin{array}{c} l_{i}=\left\|P_{i}-B_{i}\right\|,\;\left(i=1,\ldots ,6\right). \end{array}$$

The direction vector of the cylinder legs can be expressed as follows:

(7) $$\begin{array}{c} e_{i}=\frac{1}{l_{i}}\left(P_{i}-B_{i}\right)\left(i=1,\ldots ,6\right). \end{array}$$

The time derivative of formula (6) shows that the velocity equation of the legs is

(8) $$\begin{array}{c} {\dot{l}}_{i}=e_{i}\cdot \dot{p}+\left(p_{i}\times e_{i}\right)\cdot \omega_{p}. \end{array}$$

The expansion speed expression of the six actuators is combined into a matrix, as follows:

(9) $$\begin{array}{c} \dot{l}=J\left[\begin{array}{c} \dot{P}\\ \omega_{p} \end{array}\right], \end{array}$$

where *J* is the Jacobian matrix as follows:

(10) $$\begin{array}{c} J=\left[\begin{array}{cc} e_{1}^{T} & {\left(p_{1}\times e_{1}\right)}^{T}\\ \vdots & \vdots \\ e_{6}^{T} & {\left(p_{6}\times e_{6}\right)}^{T} \end{array}\right]. \end{array}$$

The expansion acceleration of the six actuators is given by the following equation:

(11) $$\begin{array}{c} \ddot{l}=\frac{\text{d}J}{\text{d}t}\left[\begin{array}{c} \dot{p}\\ \omega_{p} \end{array}\right]+J\left[\begin{array}{c} \ddot{p}\\ \omega_{p} \end{array}\right]. \end{array}$$

Given the pose parameters of the platform at a certain time, the motion speed of the driving rods of each leg of the Stewart platform can be obtained by using the inverse solution of formula (9), and the motion acceleration of each driving rod of the Stewart platform can be obtained by using formula (11).

One of the electric cylinders is considered for stress analysis, as shown in Figure 5. The force of each electric cylinder on the beam can be expressed as follows:

(12) $$\begin{array}{c} F_{i}^{c}=M_{T}\left(X{\;}^{\prime \prime }\left(t\right)+L_{T}\omega_{i}^{2}\cos\;\theta_{i}\right)+M_{G}\left(x_{Gi}^{\prime \prime }+L_{G}\omega_{i}^{2}\right)\cos\;\theta_{i},\;\left(i=1,2\ldots 6\right), \end{array}$$

where *M*_*G*_ is the mass of the electric cylinder rod, *M*_*T*_ is the mass of the electric cylinder barrel, *L*_*G*_ is the distance from the center of the mass of the electric cylinder rod to the lower joint point, *L*_*T*_ is the distance from the center of the mass of the electric cylinder barrel to the lower joint point, $\ddot{X}\left(t\right)$ is the vertical acceleration of beam vibration, and *ω*_*i*_ is the angular velocity of the electric cylinder.

The beam and the helicopter simulation cabin are connected by an inverted Stewart platform, the down-platform area of the Stewart platform is connected with the simulation cabin, and the up-platform area is connected with a trolley supported by the beam. Then, the support force provided by the beam can be expressed by *F*_*N*_ in the vertical direction, as follows:

(13) $$\begin{array}{c} F_{N}=M_{C}\left(x_{c}^{\prime \prime }+g\right)+M_{B}\left(x{\;}^{\prime \prime }\left(t\right)+g\right)+\sum_{i=1}^{6}F_{i}^{c}, \end{array}$$

where *F*_*N*_ is the support force provided by the beam in the vertical direction, *M*_*C*_ is the total mass of the simulation cabin, and *M*_*B*_ is the total mass of the upper base including the trolley and subsidiary equipment.

When the helicopter hovering rescue simulation system is in the working state, the Stewart platform drives the motion of the simulation cabin and feeds back the exciting force to the crane beam, which changes irregularly over time. With an aperiodic excitation of this kind, the system usually has no steady state but rather a transient vibration. The analysis method of the system response with irregular excitation is to decompose the aperiodic excitation force into a series of impulse loads. The system response should be superimposed by all of the impulse responses under impulse loads at different times [28].

The impulsive vibration is a free vibration with an initial velocity of 1/*m* and an initial displacement of zero [29]. When the impulsive force acts on *t*=*τ*, the vibration response of the object is as follows:

(14) $$\begin{array}{c} x\left(t-\tau \right)=\frac{1}{m\omega_{d}}e^{-\xi \omega_{n}\left(t-\tau \right)}\sin\;\omega_{d}\left(t-\tau \right), \end{array}$$

where *ω*_*n*_ is the natural frequency, *ω*_*d*_ is the decaying vibration frequency, and *ξ* is the damping coefficient.

The system can be simplified as a simply supported beam with a lumped mass, as shown in Figure 6. It is assumed that the beam is homogeneous and uniform. The lumped mass *m* is placed at the midpoint of the beam. The length of the beam is *L*, the mass per unit length is *qL*, and the bending stiffness is *EI*.

The main beam and the end beam of the crane are welded by steel plates, and the box is surrounded by an upper cover plate, a lower cover plate, and a web plate. The thickness of the steel plate is 30 mm. The internal support of the box is composed of stiffeners, diaphragms, and side bars, as shown in Figure 7.

The static deflection equation of a simply supported beam with a lumped mass is as follows:

(15) $$\begin{array}{c} y\left(x\right)=y_{s}\cdot \left[\frac{3x}{L}-4{\left(\frac{x}{L}\right)}^{3}\right],\;0\leq x\leq \frac{L}{2}, \end{array}$$

where *y*_*s*_  is the deflection at the midpoint of the crossbeam, given by the following equation:

(16) $$\begin{array}{c} y_{s}=\frac{mgl^{3}}{48EI}. \end{array}$$

Assuming that the dynamic deflection of the midpoint of the beam is *y*_*d*_, the movement process is expressed as follows:

(17) $$\begin{array}{c} y_{d}=A\;\sin\left(\omega_{n}t+\varphi \right). \end{array}$$

The dynamic deflection equation of the beam at the *x* position can be expressed as follows:

(18) $$\begin{array}{c} Y\left(x\right)=y_{d}\cdot \left[\frac{3x}{L}-4{\left(\frac{x}{L}\right)}^{3}\right],\;0\leq x\leq \frac{L}{2}. \end{array}$$

Dividing the beam into microsegments  *dx*, the total kinetic energy can be expressed as follows:

(19) $$\begin{array}{c} T=\int_{0}^{l}\frac{1}{2}\rho \cdot \dot{Y}{\left(x\right)}^{2}\text{d}x+\frac{1}{2}m\cdot {\dot{y}}_{d}^{2}. \end{array}$$

The maximum total kinetic energy of the system is given by the following equation:

(20) $$\begin{array}{c} T_{\max}=\frac{1}{2}\left(m+\frac{17}{35}\rho L\right)A^{2}\omega_{n}^{2}. \end{array}$$

The maximum potential energy of the system is given by the following equation:

(21) $$\begin{array}{c} U_{\max}=\frac{1}{2}kA^{2}, \end{array}$$

where *k* is the equivalent stiffness coefficient for the beam, *k*=*mg*/*y*_*s*_.

The maximum kinetic energy and the potential energy of the system are equal, and *U*_max_=*T*_max_ is simplified as follows:

(22) $$\begin{array}{c} \omega_{n}=\sqrt{\frac{k}{m+17/35\rho L}}. \end{array}$$

The excitation force *F*_*N*_(*t*) that acts on the beam can be regarded as a superposition of a series of impulses. For linear systems, the excitation force *F*_*N*_(*t*) can be expressed in convolution form, as follows:

(23) $$\begin{array}{c} X\left(t\right)=\int_{0}^{\tau }F_{N}\left(\tau \right)\cdot x\left(t-\tau \right)\text{d}\tau . \end{array}$$

Then, the support force provided by the beam can be expressed by substituting formulas (13) and (14) into formula (23). For the condition that the expected trajectory of the Stewart platform is known, the vibration displacement *X*(*t*) of the beam can be obtained.

### 3.2. Driving Equation of Electric Cylinder Leg

The Stewart platform has an EXLAR FT35 type turn-back electric cylinder as an outrigger. The servo motor is a model of the Phase company, a U30720A40.3BSKYZ servo motor, as listed in Table 1. The drive is a 14.F5, a 1D-34MA model of the KEB company. The electric cylinder is composed of an AC servo motor, a ball screw, and relevant transmission parts, as shown in Figure 8(a).  Figure 8(b) shows the equivalent diagram of the electric cylinder, where *u*_*e*_ is the rated voltage of the electric cylinder, *J*_*d*_ is the moment of inertia of the motor rotor, *J*_*z*_ is the moment of inertia of the load, *L*_*e*_ and *R*_*e*_ are the equivalent inductance and the equivalent resistance of the servo motor, respectively, *M*_*d*_ is the motor torque, *ω*_*d*_ is the motor speed, *i*_*z*_ is the transmission ratio, *γ* is the potential coefficient, which is related to the rated voltage of the electric cylinder and the internal coil structure, and *λ* is the torque coefficient, which is related to the rated voltage and the rated torque of the electric cylinder.

The servo motor transfer function is given by the following equation:

(24) $$\begin{array}{c} G\left(s\right)=\frac{W\left(s\right)}{U\left(s\right)}. \end{array}$$

The relationship between the voltage and the angular velocity is linear, which can be seen from the voltage balance equation:

(25) $$\begin{array}{c} U\left(s\right)=\gamma W\left(s\right)+\lambda M\left(s\right). \end{array}$$

According to the moment balance equation,

(26) $$\begin{array}{c} M\left(s\right)=J_{\sum }W\left(s\right)\cdot s+bW\left(s\right), \end{array}$$

The total moment of inertia on the motor is as follows:

(27) $$\begin{array}{c} J_{\sum }=J_{d}+\frac{J_{z}}{i_{z}^{2}\eta }. \end{array}$$

Substituting formulas (25) and (26) into formula (24) yields

(28) $$\begin{array}{c} G\left(s\right)=\frac{1}{\gamma +\lambda b+\lambda J_{\sum }s}. \end{array}$$

The first-order differential transmission model of the electric cylinder can be obtained by substituting the numerical value:

(29) $$\begin{array}{c} G\left(s\right)=\frac{1.79}{1+0.035s}. \end{array}$$

### 3.3. Vibration Controller

It is difficult to eliminate the vibration in the accurate control of Stewart platform, which is caused by the large size and heavy mass of the placed object. However, the excitation force of the Stewart platform varies irregularly over time, and the vibration of the flexible base also affects the magnitude of the exciting force in turn. Therefore, only by quantifying the exciting force and the vibration of the flexible base itself, the problem of precise control of the system can be solved.

The dynamic model of the Stewart platform is given by the following equation:

(30) $$\begin{array}{c} M\left(q\right)\ddot{q}+C\left(q,\dot{q}\right)\dot{q}+G\left(q\right)=J^{T}\Gamma , \end{array}$$

where $q,\dot{q}$, and $\ddot{q}\in R^{6}$ are the position, velocity, and acceleration of the center point of the moving platform, respectively, *M*(*q*) is the mass of the moving platform and six legs, $C\left(q,\dot{q}\right)$ is the velocity vector of the moving platform and six legs, *G*(*q*) is the gravity matrix of the moving platform and six legs, and Γ(*t*) is the output force of the six legs.

The system is controlled by a proportional derivative, and the servo rule is as follows:

(31) $$\begin{array}{c} u={\ddot{q}}_{d}-K_{v}\dot{e}-K_{p}e, \end{array}$$

where *q*_*d*_ is the desired trajectory, *e*=*q* − *q*_*d*_, $\dot{e}=\dot{q}-{\dot{q}}_{d}$, and *K*_*p*_ and *K*_*v*_ are the non-negative constant gain matrices.

The trajectory tracking control law of the Stewart Platform is as follows:

(32) $$\begin{array}{c} \Gamma \left(t\right)=J^{-T}\left[M\left(q\right)\left({\ddot{q}}_{d}-K_{v}\dot{e}-K_{p}e\right)+C\left(q,\dot{q}\right)\dot{q}+G\left(q\right)\right]. \end{array}$$

For the ideal closed-loop system model, the system error equation is as follows:

(33) $$\begin{array}{c} \ddot{e}-K_{v}\dot{e}-K_{p}e=0. \end{array}$$

Formula (36) can be written as a state-space expression, as follows:

(34) $$\begin{array}{c} \dot{X}=EX, \end{array}$$

where

(35) $$\begin{array}{c} X={\left[\begin{array}{cc} e & \dot{e} \end{array}\right]}^{T},\\ E=\left[\begin{array}{cc} o & I\\ -K_{p} & -K_{V} \end{array}\right]. \end{array}$$

According to the matrix exponential algorithm,

(36) $$\begin{array}{c} X=e^{Et}X\left(0\right). \end{array}$$

By selecting reasonable parameters for *K*_*p*_ and *K*_*v*_, we can obtain the formula $\underset{t⟶\infty }{\lim}e\left(t\right)=0$.

The dynamic coupling compensation model of the helicopter hovering rescue simulation system is shown in Figure 9. Before the expected trajectory of the engine room motion is input to the Stewart platform, the compensation parameter *X*(*t*) is solved through the solution of the dynamic coupling compensation model. After the compensation amount compensates for the desired trajectory in real time, through the dynamic inverse solution of the Stewart platform, the output of six electric cylinders is the extension, which is input to the Stewart platform after PD control to achieve the real-time and accurate control of the system, If the dynamic model is accurate, the compensation model can achieve dynamic decoupling. Referring to Section 3.1, the dynamic coupling algorithm module includes two parts: one part is the excitation force solution module and the other part is the random response solution module. The excitation force solution module calculates the initial excitation force with the expected trajectory of the engine room as the initial value. Through the dynamic solution of the Stewart platform, the instantaneous excitation force acting on the flexible base is output to the random response solution module. The random response solution module is used to calculate the expected vibration response of the beam based on the parameters of the crane beam, and then, the parameter value of the expected vibration response is fed back to the excitation force solution module for real-time correction calculation.

## 4. Results

### 4.1. Experimental System

The experimental system of the helicopter rescue simulator based on the flexible base is shown in Figure 10. The transverse beam of the crane is 37.4 m long, and this beam is welded into a box by the upper cover plate, the lower cover plate, and the web plate. The thickness of the steel plate is 30 mm, and the internal support of the box is composed of stiffeners, diaphragms, and side bars. The beam material is Q235B, and its performance parameters are a density of 7.85 × 10^3^ kg/m^3^, a yield strength of 235 MPa, a tensile strength of 400 MPa, an elastic modulus of 2.06 × 10^5^ MPa, and a Poisson's ratio of 0.3.

The Stewart platform parameters are as follows: the maximum stroke of the leg is 440 mm and the control accuracy is 2 *µ*m. The three-axis translation range of the platform is ±400 mm, and the rotation range is ±20°. The platform has an industrial computer installed with a Labview real-time operating system as the controller, as shown in Figure 10(b). After the desired trajectory is solved with the antivibration controller, the PCI (peripheral component interconnection) motion control card outputs the data to the Stewart platform to control the action of the platform legs. At the same time, the encoder of the platform legs feeds back the movement information of the legs to the industrial computer to achieve semi-closed loop control. A new acceleration acquisition system is added on the lower platform, and the acceleration sensor (model: lc352c33) is placed at the center of the hinge circle under the platform, which is responsible for collecting the motion data of the cabin, as shown in Figure 10(c).

### 4.2. Control Experiment

The simulator is driven to the middle of the beam, and a 20-s 6-DOF position signal is input to the simulator. This signal is from a section of the helicopter hovering signal during rescue training. In the traditional PID control mode [30], the acceleration signal of the cabin is measured as curve B. In the hybrid compensation control mode, the acceleration signal of the cabin is measured as curve C. Curves B and C are compared with the desired acceleration signal curve A to obtain the experimental results that are shown in Figure 11. To make the display clearer, 4–5 s and 19–20 s of the curves are considered for comparison. It can be seen that curve B cannot follow curve A well, and it shows that single PID control cannot solve the vibration interference problem of flexible base; curve C has a better coincidence compared to curve B with curve A. It is proven that the vibration compensation control has a better compensation effect than the traditional PID control. It is effective to solve the problem of precise control for the flexible base that has a large range of motion [31].

## 5. Conclusions

The traditional Stewart control methods are mostly based on a rigid base. For large flexible parts, the control method of actively suppressing the vibration of flexible parts is also not ideal. For the special application of the crane beam of a helicopter rescue simulator, which has large flexible parts, violent vibration, and a large range of motion, this study establishes the dynamic model of a Stewart platform, considering beam vibration. The experimental results show that the model has a good antivibration effect. This method has good application prospects in situations where the installation of the motion acquisition system is difficult and the flexible parts are large in size.

## Figures and Tables

**Figure 1:** The helicopter hovering rescue system.

**Figure 2:** Components of the helicopter hovering rescue simulator. 1. Trolley. 2. Stewart platform. 3. Electric winch. 4. Bridge crane beam. 5. Helicopter simulation cabin.

**Figure 3:** Vibration of the beam during a training process.

**Figure 4:** Structure parameters of inverted Stewart platform.

**Figure 5:** Velocity vector diagram of electric cylinder.

**Figure 6:** The beam with lumped mass.

**Figure 7:** Box structure of the beam. 1. Partition. 2. Reinforcement. 3. Square steel track. 4. Stiffener.

**Figure 8:** Structure of the electric cylinder leg. (a) Mechanical schematic of the electric cylinder. (b) Equivalent diagram of the electric cylinder.

**Figure 9:** Vibration hybrid controller schematic.

**Figure 10:** Experimental equipment of helicopter rescue simulator. (a) Schematic diagram of the experiment. (b) Experimental system. (c) Position of Acceleration Sensor.

**Figure 11:** Acceleration signal of the cabin during a training task.

**Table 1:** Specification parameters of the electric cylinder.

Symbol	Physical sense	Value and unit
*γ*	Potential coefficient	0.53 V∙s/rad
*λ*	Torque coefficient	8.87 V∙m/N
*J*_*d*_	Moment of inertia of the motor rotor	0.0004 kg∙m^2^
*J*_*z*_	Moment of inertia of the load (screw)	0.0016 kg∙m^2^
*i*_*z*_	Transmission ratio	1 : 1
*η*	Transmission efficiency	0.9
*b*	Equivalent viscous friction coefficient	0.003 N∙s/m

## Data Availability

The dataset used in this paper is available from the corresponding author upon request.
